# A Blind Watermarking Model of the 3D Object and the Polygonal Mesh Objects for Securing Copyright

**DOI:** 10.1155/2021/1392903

**Published:** 2021-11-30

**Authors:** Hanan S. Al-Saadi, A. Ghareeb, Ahmed Elhadad

**Affiliations:** ^1^Department of Mathematics, Faculty of Applied Sciences, Umm Al-Qura University, Makkah, Saudi Arabia; ^2^Department of Mathematics, Faculty of Science, Al-Baha University, Al Bahah, Saudi Arabia; ^3^Department of Mathematics, Faculty of Science, South Valley University, Qena, Egypt; ^4^Department of Computer Science, Faculty of Computers and Information, South Valley University, Qena, Egypt; ^5^Computer Science and Information Department, College of Science and Arts, Jouf University, Sakakah, Saudi Arabia

## Abstract

In this paper, we propose a novel model for 3D object watermarking. The proposed method is based on the properties of the discrete cosine transform (DCT) of the 3D object vertices to embed a secret grayscale image three times. The watermarking process takes place by using the vertices coefficients and the encrypted image pixels. Moreover, the extraction process is totally blind based on the reverse steps of the embedding process to recover the secret grayscale image. Various performance aspects of the method are measured and compared between the original 3D object and the watermarked one using Euclidean distance, Manhattan distance, cosine distance, and correlation distance. The obtained results show that the proposed model provides better performances in terms of execution time and invisibility.

## 1. Introduction

Recently, browsing online is an imperative portion of our life so digital data and objects are easy to be duplicated by users to make unauthorized and fake copies of the original work. All kinds of digital data and objects have intellectual-property protection from the owner which is called copyrights. Therefore, copyright is the exclusive legal right of the owner that gives him the right to make copies of creative work, literary, and artistic works. In digital media, the creative work, literary, and artistic works refer to digital objects such as e-books, images, videos, music, databases, and 3D objects. Intensively, the 3D objects are utilized in various purposes such as games, computer graphics, medical imaging, manufacturing, and human models. Thus, the copyright of the 3D object needs more requesting to push research towards developing protection techniques. Watermarking is one of the most important proposed solutions for intellectual-property protection of the 3D object. For securing copyright, the watermark must be robust against the unauthorized use.

In modern times, watermarking techniques for a wide range of digital media were utilized as a host cover to hide or embed a piece of information message in such a way that it is imperceptible to a human observer. Usually, the digital media covers can take any form such as images [1–7], videos [8–12], audio [13–15], and DNA sequences [16, 17]. Even so the 3D objects are widely available and important, there are a few existing watermarking techniques. The various watermarking techniques for 3D objects can be classified according to the embedding domains such as the spatial domain [18, 19], the spectral-domain [20, 21], and the transform domain [22, 23]. The transform domain techniques such as Fourier, Laplace, cosine, and wavelet transform provide a good trade-off between invisibility and robustness.

In this paper, we propose a novel model for 3D object watermarking. The proposed method is based on the properties of the discrete cosine transform (DCT) of the 3D object vertices to embed a secret grayscale image three times. Different performance aspects of the method are measured and compared between the original 3D object and the watermarked one. The rest of the paper is organized as follows.  Section 2 gives a related work on data hiding and watermarking in 3D objects.  Section 3 describes the watermarking model of the proposed technique. Experimental results are presented and analyzed in Section 4, where a performance comparison was held between the original 3D object and the watermarked object. Finally, Section 5 summarizes the findings and conclusions.

## 2. Related Work

In [24], Ai et al. proposed a 3D triangular mesh models watermarking scheme. The proposed method was based on selecting the significant geometry information of triangular meshes. Then, the watermark bits are repeatedly embedded into the corresponding Voronoi patch using the high frequency coefficients of the discrete cosine transform. The advantages of the proposed method are resistant to common attacks and provide good imperceptibility. Based on the graph Fourier transform in [22], Ferreira et al. proposed a nonblind 3D point cloud watermarking method. The proposed method assumes the points of connectivity information to represent the cloud as a graph. Then, the watermark bits are embedded in the spectral graph of the Fourier domain. Similarly, in [25], the authors presented a robust 3D point cloud models watermarking in spatial domain. In [26], Zhang et al. presented a 3D geological model watermarking algorithm based the principal component analysis of the point cloud model of geological body.

In [27], El Zein et al. presented two 3D watermarking schemes based on fuzzy c-means clustering technique in the spatial domain. The proposed methods start by selecting the appropriate vertices using the fuzzy c-means clustering using the feature vector. Then, the watermark bits are embedded into the selected vertices using two insertion methods based on statistical measurements. The first method achieved higher results in robustness while the second method achieved higher results in imperceptibility. In the same context in [23], Liu et al. proposed the blind and robust 3D object watermarking method based on the multiresolution adaptive parameterization of surface approach for vertices classification. The results of the proposed method showed that it has good imperceptibility and it resists to common attacks. Moreover in [28, 29], Medimegh et al. presented a statistical 3D object watermarking method based on extracting the salient feature points using autodiffusion function. The proposed method segments the 3D object into regions according to the salient points, and then it inserts the watermark bits using the embedding method in [30].

In [31], Molaei et al. proposed a fragile and blind watermarking method based on the geometrical properties of the 3D object. The proposed method selects a specific triangular and embeds the watermark bit using the medians of the triangular faces in spherical coordinates and reconstructs a new triangle. Based on the geometric property of vertices in [32], Hansda et al. proposed a nonblind method to watermark the 3D object using the mean curvature of vertices. The method divided the vertices into two groups: the first group includes the convex curvature vertices and the second group is the rest of vertices. Then, the watermark bits are embedded by modifying the vertices using the first group. Instead of using the geometric distortions, in [33], Son et al. presented a blind 3D object watermarking method based on mesh saliency. The proposed method uses the distribution of the vertex norm histogram and combines between the spatial domain embedding and the frequency-based weight map.

Based on the above, the main contributions of this paper are as follows: (1) we introduce a 3D object watermarking scheme that takes advantage properties of the discrete cosine transform (DCT) to hide a grayscale image into the 3D object vertices; (2) we propose a blind extraction based on the reverse steps of the embedding process to recover the secret grayscale image; (3) we brought evidence that the proposed watermarking scheme performed across the different 3D objects ensures a minimum shape distortion; and (4) we present comprehensive experimentation examining the performance of our method and comparing it with other methods.

## 3. The Proposed Model

The 3D object watermarking means adding integrated hidden information into polygonal mesh object without leaving visual marks or causing any structural changes. It is typically used to identify ownership rights of such that original 3D object and protect it from theft. In this inevitable scenario, in this paper, there is a proposed method for watermarking the 3D object, which takes advantage properties of the discrete cosine transform (DCT) to hide a grayscale image into the 3D object vertices.

Figure 1 depicts the overall process of the proposed watermarking model. Firstly, the proposed method normalizes both the original 3D object vertices and the secret grayscale image. This step allows us to apply the appropriate fuzzy algorithms for modifying the membership values. In general, there are different approaches to fuzzification and many applications such as [34, 35]. Then, a preprocessing is applied on the normalized 3D object vertices and applies a discrete cosine transform (DCT) for every three vertices. In the same time, reshape and encryption processes are carried out on the normalized watermark image. After that, the watermarking process will take place by using the vertices coefficients and the encrypted image pixels. Finally, the inverse DCT and denormalization process of the modified vertices will be applied to produce the watermarked 3D object.

### 3.1. The Embedding Procedure

As mentioned above, the process of embedding the watermark starts by normalizing both the original 3D object vertices and the secret grayscale image. Generally, normalization is a typical process that expands the range of data values dynamically. Therefore, normalization changes the data object Obj :  {*X* ⊆ℝ^*d*^}⟶{Min,…,  Max} from the range values [Min, Max] into a new data object Obj_New_ :  {*X* ⊆ℝ^*d*^}⟶{Min_New_,…, Max_New_} with the range values [Min_New_, Max_New_]. The linear normalization of a data object is performed according to the following formula:

(1) $$\begin{array}{c} {\text{Obj}}_{\text{New}}=\left(\text{Obj}-\text{Min}\right)\frac{{\text{Max}}_{\text{New}}-{\text{Min}}_{\text{New}}}{\text{Max}-\text{Min}}+{\text{Min}}_{\text{New}}. \end{array}$$

In the proposed method, the normalization process refers to change both the original 3D object vertices and the secret grayscale image data range with intensity values in the range of [0,1]. So, the normalization is achieved according to the following formula:

(2) $$\begin{array}{c} {\text{Obj}}_{\text{New}}=\frac{\left(\text{Obj}-\text{Min}\right)}{\text{Max}-\text{Min}}. \end{array}$$

For security issue, the secret grayscale image is encrypted using the seed numbers of a pseudorandom generator, and this scrambles the position of every pixel in the original grayscale image. The encryption process is applied to the reshaping to vector of the grayscale image to increase the complexity of the scrambling. In addition, it changes the position of the pixels using three secret keys to provide better robustness in this system.

In the preprocessing phase, the normalized vertices of the original 3D object are adjusted using *α* :  (*α* ∈ ℝ, 0 < *α* ≪ 1). This phase assures that saturated vertex value would not eventually result in an overflow in the embedded vertex coefficient. So, the preprocessing phase takes place according to the following formula:

(3) $$\begin{array}{c} 3D\text{ Obj}\left(\text{Vertex}\right)=\left\{\begin{array}{cc} \alpha , & \text{Vertex}=0,\\ 1-\alpha , & \text{Vertex}=1. \end{array}\right. \end{array}$$

The discrete cosine transform (DCT) is derived from the Fourier-related transformation [36], and Ahmed et al. firstly proposed the discrete cosine transform (DCT) in [37]. DCT transforms a sequence of real data points into its real spectrum to avoid the problem of redundancy. Thus, the DCT is the process of decomposing a finite sequence of digital signal data points in terms of a sum of cosine functions oscillating at different frequencies to be the equivalent of the original digital signal. Formally, the DCT is an invertible function *f*  : *ℝ*^*d*^⟶ *ℝ*^*d*^, so for a signal *x* of length *N* and with *δ* the Kronecker delta, the DCT has four standard variants according to one of the following formulas.

The type DCT-1:

(4) $$\begin{array}{c} y\left(k\right)=\sqrt{\frac{2}{N-1}}\sum_{n=1}^{N}x\left(n\right)\frac{1}{\sqrt{1+\delta_{n1}+\delta_{nN}}}\frac{1}{\sqrt{1+\delta_{k1}+\delta_{kN}}}\cos\left(\frac{\pi }{2N}\left(n-1\right)\left(k-1\right)\right). \end{array}$$

The type DCT-2:

(5) $$\begin{array}{c} y\left(k\right)=\sqrt{\frac{2}{N}}\sum_{n=1}^{N}x\left(n\right)\frac{1}{\sqrt{1+\delta_{k1}}}\cos\left(\frac{\pi }{2N}\left(2n-1\right)\left(k-1\right)\right). \end{array}$$

The type DCT-3:

(6) $$\begin{array}{c} y\left(k\right)=\sqrt{\frac{2}{N}}\sum_{n=1}^{N}x\left(n\right)\frac{1}{\sqrt{1+\delta_{n1}}}\cos\left(\frac{\pi }{2N}\left(n-1\right)\left(2k-1\right)\right). \end{array}$$

The type DCT-4:

(7) $$\begin{array}{c} y\left(k\right)=\sqrt{\frac{2}{N}}\sum_{n=1}^{N}x\left(n\right)\cos\left(\frac{\pi }{4N}\left(2n-1\right)\left(2k-1\right)\right), \end{array}$$

where

(8) $$\begin{array}{c} k=0,1,\;\ldots ,N,\\ \delta_{ij}=\left\{\begin{array}{cc} 0, & \text{if }i\neq j,\\ 1, & \text{if }i=j. \end{array}\right. \end{array}$$

The proposed method supposes that the 3D object has *L* set of vertices, and each vertex is defined as Vertex(*X*, *Y*, *Z*). Thus, the next phase is applying the DCT transform for each vertex as a vector using the following formula:

(9) $$\begin{array}{c} f\left(\text{Vertex}\left(X_{l},Y_{l},Z_{l}\right)\right)⟶\left({\text{Coefficient}}_{1l},{\text{Coefficient}}_{2l},{\text{Coefficient}}_{3l}\right),\\ \forall \left(\text{Vertex}\left(X_{l},Y_{l},Z_{l}\right)\right),\;l=1,\;2,\ldots ,L. \end{array}$$

Once the DCT is applied on the normalized 3D object vertices, the next step carries out the watermarking process on the normalized coefficients of the vertices. Therefore, the first coefficient value will be within the interval [0, 2], and the values of the second and the third coefficient will be within the interval [−1, 1]. Using these facts, we construct the following equation system for watermarking the secret grayscale image in the transformed regions of the 3D object coefficients:

(10) $$\begin{array}{c} 3D\text{ obj}\left(\hat{C}\right)=\frac{2}{\beta }\left(\text{EncMsg}+i\right)\;,\\ \frac{2i}{\beta }\leq 3D\text{ obj}\left(C\right)<\frac{2\left(i+1\right)}{\beta },\\ i=\left\{\begin{array}{cc} 0,\;1,\;2,\;3,\ldots ,\left(\beta -1\right), & C=\left\{{\text{Coefficient}}_{1}\right\},\\ -2,-1,0,1,\ldots ,\left(\beta -3\right), & C=\left\{{\text{Coefficient}}_{2},{\text{Coefficient}}_{3}\right\}, \end{array}\right. \end{array}$$

where in these equation system, $3\;D\text{ obj}\left(\hat{C}\right)$ refers to the current coefficient in the watermarked 3D object vertices, 3  *D* obj(*C*) is the corresponding coefficient in the 3D object vertices, EncMsg is the embedded pixel in the secret grayscale image, and *β* is the number of intervals which satisfy that the coefficient on the interval of [0, 2] or [–1, 1] corresponding to the coefficients *C*. Finally, the inverse of the DCT transform and denormalization process are used to reconstruct the watermarked 3D object with the secret embedded grayscale image. Full details of the embedding process are shown with the mathematical relationships contained as pseudocode in Algorithm 1.

### 3.2. The Extraction Procedure

In the extraction process, the steps carried out in the embedding process are generally reversed to recover the secret grayscale image. The steps of the extraction module are illustrated in Figure 2. Thus, the process starts by normalizing the watermarked 3D object and then computing the DCT transform decomposition of the vertices. So, the encrypted grayscale image pixel can be extracted using the parameters *β* and the $3\;D\text{ obj}\left(\hat{C}\right)$ coefficients according to the following equation:

(11) $$\begin{array}{c} \text{EncMsg}=\frac{\beta }{2}\left(3D\text{ obj}\left(\hat{C}\right)-\frac{2i}{\beta }\right)\text{,}\\ \;\frac{2i}{\beta }\leq 3D\text{ obj}\left(\hat{C}\right)\leq \frac{2\left(i+1\right)}{\beta },\\ i=\left\{\begin{array}{cc} 0,\;1,\;2,\;3,\ldots ,\left(\beta -1\right), & \hat{C}=\left\{{\text{Coefficient}}_{1}\right\},\\ -2,-1,0,1,\ldots ,\left(\beta -3\right), & \hat{C}=\left\{{\text{Coefficient}}_{2},{\text{Coefficient}}_{3}\right\}. \end{array}\right. \end{array}$$

In blind manner and using *β*, the secret EncMsg will be extracted from the watermarked 3D object. Next, the three keys are required to identify the position at which the secret original pixels were located. Since the pixel values were normalized, they need to be denormalized to convert the pixel values back to their original integer domain. Notice that the secret grayscale image is extracted correctly three times. The full details of the extraction part are displayed as pseudocode in Algorithm 2.

## 4. Experimental Results and Discussion

### 4.1. Implementation

Throughout the following sets of experiments, Figures 3(a)to 3(f) show six standard 3D objects which were used for testing the proposed method performance. In addition, Figure 3(g) shows the secret grayscale image which was used as watermark image in size of 114 × 57, 315 × 128, 597 × 349, 615 × 473, 1119 × 453, and 1728 × 823. The proposed model was implemented using Intel(R) Core (TM) i7-4700MQ CPU, 2.40 GHz processor with 8 GB of RAM. Moreover, the MATLAB version 9.0.0.341360 (R2016b) was used in coding the implementation. In the encryption step, three seeds for the random number generator were selected to be 1987, 1989, and 1993.

In the field of data hiding, techniques are compared according to several parameters such as capacity and payload. The definition of capacity is that the maximum bits hidden within the 3D object vertices. The actual payload is the percentage between the current embedded bits and the capacity of the 3D object in bits.  Table 1 presents the resultant capacity and the actual payload for each 3D object and the corresponding embedded secret grayscale image. That is, given *L* vertices in the original 3D, so the capacity in bits per vertex (bpv) and the actual payload in percent (*%*) can be computed as the following:

(12) $$\begin{array}{c} \text{capacity}=\;\frac{\text{Max}\left(\text{number of embedded pixels}\right)\times 8}{\text{number of vertices}}=\;\frac{L\times 8}{L}\;=8\text{ bpv},\\ \text{actual payload}=\;\frac{\text{secret image size in bits}\times 3\times 100}{3D\text{ object capacity in bits}}. \end{array}$$

Figure 4 shows the experiments and time taken to watermark and extract the maximum capacity for each 3D object and values of *β* between 1000 and 9000 to evaluate the time performance of the proposed method. Obviously, the extraction execution time is less than the watermarking execution time for the same 3D object. Thus, the average time performance is 3.11, 18.72, 94.56, 133.19, 227.15, and 636.90 seconds for watermarking process the Glock, egg, bunny, horse, cat, and angel models, respectively. In the same context, the average time performance for the extraction process is 1.99, 12.19, 60.98, 86.83, 146.38, and 406.65 seconds for the Glock, egg, bunny, horse, cat, and angel models, respectively. Obviously, the parameter *β* has a very little effect on the time execution for the same 3D object.

The imperceptibly and the transparency performances of the proposed method were evaluated using Euclidean distance, Manhattan distance, cosine distance, and the correlation distance. Let the original 3D object be *u* and the watermarked object be *v*, the invisibility performance term details were explained in the following equations.

The Euclidean distance is as follows:

(13) $$\begin{array}{c} \text{Euclidean dist}\left(u,v\right)=\sqrt{{\left|u_{x}-v_{x}\right|}^{2}+{\left|u_{y}-v_{y}\right|}^{2}+{\left|u_{z}-v_{z}\right|}^{2}}. \end{array}$$

Manhattan distance is as follows:

(14) $$\begin{array}{c} \text{Manhattan dist}\left(u,v\right)=\left|u_{x}-v_{x}\right|\;+\left|u_{y}-v_{y}\right|+\left|u_{z}-v_{z}\right|\text{ .} \end{array}$$

Cosine distance is as follows:

(15) $$\begin{array}{c} \text{cosine dist}\left(u,v\right)=1-\frac{u_{x}v_{x}+u_{y}v_{y}+u_{z}v_{z}}{\sqrt{{\left|u_{x}\right|}^{2}+{\left|u_{y}\right|}^{2}+{\left|u_{z}\right|}^{2}}\sqrt{{\left|v_{x}\right|}^{2}+{\left|v_{y}\right|}^{2}+{\left|v_{z}\right|}^{2}}}. \end{array}$$

The correlation distance is as follows:

(16) $$\begin{array}{c} \text{correlation dist}\left(u,\;v\right)\;=\;1-\frac{\left(\left(1/3\right)\left(-u_{x}-u_{y}-u_{z}\right)+u_{x}\right)\left(\left(1/3\right)\left(-v_{x}-v_{y}-v_{z}\right)+v_{x}\right)+\left(\left(1/3\right)\left(-u_{x}-u_{y}-u_{z}\right)+u_{y}\right)\left(\left(1/3\right)\left(-v_{x}-v_{y}-v_{z}\right)+v_{y}\right)+\left(\left(1/3\right)\left(-u_{x}-u_{y}-u_{z}\right)+u_{z}\right)\left(\left(1/3\right)\left(-v_{x}-v_{y}-v_{z}\right)+v_{z}\right)}{\sqrt{{\left|u_{x}+\left(1/3\right)\left(-u_{x}-u_{y}-u_{z}\right)\right|}^{2}+{\left|u_{y}+\left(1/3\right)\left(-u_{x}-u_{y}-u_{z}\right)\right|}^{2}+{\left|\left(1/3\right)\left(-u_{x}-u_{y}-u_{z}\right)+u_{z}\right|}^{2}}\sqrt{{\left|v_{x}+\left(1/3\right)\left(-v_{x}-v_{y}-v_{z}\right)\right|}^{2}+{\left|v_{y}+\left(1/3\right)\left(-v_{x}-v_{y}-v_{z}\right)\right|}^{2}+{\left|\left(1/3\right)\left(-v_{x}-v_{y}-v_{z}\right)+v_{z}\right|}^{2}}}. \end{array}$$

Figure 5 shows the obtained Euclidean distance, Manhattan distance, cosine distance, and the correlation distance result to compare between the original 3D object and the resultant watermarked using values of *β* between 1000 and 9000. Moreover, the experiments investigate the effect of the embedding parameters *β* on the fidelity of the embedding when applying the maximum capacity. The average resultant Euclidean distance for Glock, egg, bunny, horse, cat, and angel objects is 30.73, 41.14, 77.62, 54.22, 75.48, and 78.16, respectively. The average resultant Manhattan distance for Glock, egg, bunny, horse, cat, and angel objects is 7.29*E* + 03, 1.42*E* + 04, 2.87*E* + 04, 1.77*E* + 04, 2.76*E* + 04, and 2.29*E* + 04, respectively. The average resultant cosine distance for Glock, egg, bunny, horse, cat, and angel objects is 0.0006, 0.0008, 0.0032, 0.0014, 0.0038, and 0.0030, respectively. The average resultant correlation distance for Glock, egg, bunny, horse, cat, and angel objects is 0.02, 0.02, 0.09, 0.06, 0.10, and 0.22, respectively. The obtained results show that *β* provides better invisibility performances of the watermarked object for large values in various terms.

The main characteristics comparison of the proposed method with other existing methods are introduced to confirm its validity and efficiency. The comparative study is conducted in order to verify the used cover media, the watermark sequence, the embedding space, the domain, the capacity, and the blindness extraction process between the proposed method and other methods.  Table 2 shows a comparison of the recorded details of the related methods. In [38–41], the presented methods were based on embedding the QR code and binary bits into images based on various domains. Moreover, Ayubi et al. in [12] presented a video watermarking method using 2D binary image. On the other hand, in [42, 43], the proposed methods watermarked the 3D printed object, and in [18, 44–46], the presented methods were based on watermarking the 3D object using a different watermark sequence. The capacities are recorded by the number of bits per pixel (bpp) and the number of bits per vertex (bpv). The proposed 3D mesh watermarking technique achieves the advantage characteristic of using high-capacity number of bits per vertices. On the contrary, watermarking schemes for copyright protection target the shape and their capacity are usually a fewer number of bits.

## 5. Conclusions

In this paper, a novel model for 3D object watermarking was proposed. The proposed method is based on the properties of the discrete cosine transform (DCT) of the 3D object vertices to embed a secret grayscale image three times. The extraction process is totally blind based on the reverse steps of the embedding process to recover the secret grayscale image. The proposed model was implemented using MATLAB, and the time performance of the proposed method was recorded. The resultant maximum capacity of the proposed method for each 3D object and the corresponding embedded secret grayscale image is 8 bits per vertex (bpv). The imperceptibly and the transparency performances of the proposed method were evaluated using Euclidean distance, Manhattan distance, cosine distance, and the correlation distance.

## Figures and Tables

**Figure 1:** The overall model for the proposed watermarking method.

**Figure 2:** The extraction flowchart of the proposed model.

**Figure 3:** The 3D objects used in the implementation and the watermark image.

**Figure 4:** The watermarking and extraction time performance of the proposed method: (a) watermarking time; (b) extraction time.

**Figure 5:** The invisibility performance of the proposed method: (a) Eulidean distance; (b) cosine distance; (c) Manhattan distance; (d) correlation distance.

**Algorithm 1:** Embedding function in the proposed method

**Algorithm 2:** Extraction function in the proposed method

**Table 1:** Embedding capacity results.

Model	Vertices	Faces	Secret image size (pixel)	Max capacity (bits)	Actual payload (%)
Glock 3D model	6564	2188	114 × 57	157536	98.995
Egg 3D model	40320	13440	315 × 128	967680	100
Stanford bunny	208353	35947	597 × 349	5000472	100
Horse	290898	48485	615 × 473	6981552	99.999
Cat figurine	506910	168970	1119 × 453	12165840	99.999
Angel	1422144	237018	1728 × 823	34131456	100

**Table 2:** Comparison of recent schemes.

Scheme	Cover media	Watermark sequence	Embedding color space	Domain	Capacity	Is blind?
Chow et al. [38]	Grayscale image	QR code	Grayscale	DWT-DCT	0.0002	Yes
Amini et al. [40]	Grayscale image	Binary bits	Grayscale	DWT	0.0156	Yes
Rosales-Roldan et al. [39]	Color image	QR code	YCbCr	SVD-DWT-DCT	0.0833	Yes
Patvardhan et al. [41]	Color image	QR code	YCbCr	SVD-DWT	0.1667	No
Ayubi et al. [12]	Video	2D binary image	RGB	IWT-DWT-CT	0.0034	Yes
Hou et al. [42]	3D printed object	Binary pattern	High masking regions	Visual masking	1 bit	Yes
Delmotte et al. [43]	3D printed object	Binary bits	G-code	Layer thickness	>64 bits	Yes
Jiang et al. [44]	3D object	Binary bits	Vertices	Encrypted domain	0.3692	Yes
Cayre et al. [45]	3D object	Binary bits	Vertices	Spatial	0.8772	Yes
Wu et al. [46]	3D object	2D binary image	Vertices	Spatial	0.9969	No
Khalil et al. [18]	3D object	Grayscale image	Vertices	Spatial	2.6667	Yes
The proposed	3D object	Grayscale image	Vertices	DCT	8	Yes

## Data Availability

The data used to support the findings of this study are included within the article.
